# Questioning the HIV-AIDS Hypothesis: 30 Years of Dissent

**DOI:** 10.3389/fpubh.2014.00154

**Published:** 2014-09-23

**Authors:** Patricia Goodson

**Affiliations:** ^1^Department of Health & Kinesiology, Texas A&M University, College Station, TX, USA

**Keywords:** HIV, AIDS, dissent, causation, multifactorial causality

Since 1984, when the hypothesis that HIV-causes-AIDS was announced, many scholars have questioned the premise and offered alternative explanations. Thirty years later, competing propositions as well as questioning of the mainstream hypothesis persist, often supported by prominent scientists. This article synthesizes the most salient questions raised, alongside theories proposing non-viral causes for AIDS. The synthesis is organized according to four categories of data believed to support the HIV-AIDS hypothesis: retroviral molecular markers; transmission electron microscopy (EM) images of retroviral particles; efficacy of anti-retroviral drugs; and epidemiological data. Despite three decades of concerted investments in the mainstream hypothesis, the lingering questions and challenges synthesized herein offer public health professionals an opportunity to reflect on their assumptions and practices regarding HIV/AIDS.

“The HIV/AIDS hypothesis is one hell of a mistake”, wrote Kary Mullis in 1996 [(1), p. 14]. Mullis – Nobel Laureate in Chemistry, 1993 – and other distinguished scientists have claimed the HIV-causes-AIDS hypothesis is false, unproductive, and unethical. They have done so since 1984, when the hypothesis was proposed. Thirty years after countless studies, resources, and attempts to cure have been poured into the HIV-AIDS hypothesis, it may be fruitful to ask: What happened to those views and voices that once disagreed? Have the past three decades, with their scientific, technological, and public health developments, been sufficient to convince critics of the hypothesis’ value? Have these advances been able to silence the questioning?

Here, I synthesize the main criticisms aimed at the HIV-AIDS hypothesis, alongside select unorthodox^1^ theories proposing non-viral cause(s) for AIDS, to argue: far from being condemned to extinction, competing explanations for, and thorough questioning of the mainstream premise persist. Perhaps better known by the lay public than by health professionals, many explanations are, in fact, attracting a growing number of sympathizers. To support the argument, I employ historical research and data synthesis methods. I utilize, as data, trade and professional publications in tandem with authoritative scientific sources.

It is important to note that my purpose is not to review the state of the science regarding HIV/AIDS, nor to persuade readers to reject the mainstream hypothesis. Instead, I aim to expose readers to the persisting controversies, and to motivate them to raise questions of their own. Ultimately, then, this article invites the public health workforce to reflect on prevailing assumptions and practices regarding HIV-AIDS. Reflecting on assumptions and practices represents a central task for public health professionals; a vital step to ensure their (our) practice continually grounds itself in the most rigorous ethical standards (3).

## HIV-Causes-AIDS: How Valid are the DATA?

In 1984, Margaret Heckler (then Secretary of the Department of Health and Human Services) announced a retrovirus was the “probable cause” of the alarming immune system collapse emerging in the US since 1981 (4). When scientists identified antibodies to a retrovirus known as LAV, or HTLV-III, in 48 persons (from a sample of 119, with and without immune deficiency symptoms), the retrovirus became the culprit of what would be perceived as “the most urgent health problem facing the country” in recent history [(5, 6), p. 1].

The announcement intended to assure the public: the mystery surrounding this apparently contagious and decidedly fatal illness – later labeled AIDS for acquired immune deficiency syndrome – was solved. The newly identified virus – soon renamed HIV, for human immunodeficiency virus – was, almost certainly, responsible for debilitating people’s immune system and making them vulnerable to infections which, before AIDS, were either rare or not particularly dangerous. Now, however, infections such as Kaposi’s Sarcoma and *Pneumocistis carinii* Pneumonia had morphed into vicious killers (4, 6). By identifying the perpetrator, scientists’ attention and government resources could then focus on treatment, cure, and vaccine development.

Yet almost immediately, scientists who knew a great deal about retroviruses and immunology began to voice misgivings regarding the HIV-causes-AIDS hypothesis, and to question it. They highlighted the difficulties, flaws, and contradictions they saw in the hypothesis, and offered alternative explanations. Many of the original misgivings have survived, and others have been raised, in the past three decades.

In this paper, therefore, I summarize some of these difficulties, and present what critics propose as alternative causes of AIDS. I organize the challenges put forth by unorthodox scholars into four categories of data that support the HIV-AIDS hypothesis^2^ : (1) retroviral molecular markers; (2) transmission electron microscopy (EM) images of retroviral particles; (3) efficacy of anti-retroviral (ARV) drugs; and (4) epidemiological data (7, 8). Because these data are proffered as solid evidence for HIV’s role in causing AIDS, it is useful to examine how critics question the evidence in each category, specifically.

### Retroviral molecular markers

Mainstream scientists and physicians claim the molecular evidence for HIV-as-the-cause-of-AIDS is irrefutable (8, 9) and comprises: (a) HIV antibodies and (b) viral load. As incontrovertible as these molecular markers appear to be, unorthodox scientists have meticulously examined each one and detected significant problems in both (7).

#### HIV antibodies

The first available tests to screen blood banks for HIV detected HIV antibodies (10). Physicians still use these tests when screening blood for infection and, since 2004, direct-to-consumer home tests have become available for identifying antibodies to HIV using only a saliva sample (e.g., OraQuick) (11). Yet, from the time the first tests appeared, scientists in both orthodox and unorthodox camps reiterated that, according to established immunology principles, antibodies to a virus indicate the immune system has acted to control the invading virus. Antibodies point to previously occurring infection and do not signal active infection. In 1984, CDC scientists (mainstream) wrote:

A positive test for most individuals in populations at greater risk of acquiring AIDS will probably mean that the individual has been infected at some time with HTLV-III/LAV [the names originally used for HIV]. Whether the person is currently infected or immune is not known, based on the serologic test alone [(12), p. 378].

It is not only this simple argument – antibodies suggest the immune system has controlled the invading agents – that unorthodox scientists have debated. The tests themselves remain the target of critic’s intense scrutiny. For instance, in 1996 Johnson reported 60-plus factors capable of causing a false-positive result on tests for HIV antibodies [either an ELISA or a western blot (WB) test] (13). Because they react to these factors, the tests may not be detecting HIV at all. Worthy of notice, among the list, are elements ubiquitous among all populations such as the flu, flu vaccinations, pregnancy in women who have had more than one child, tetanus vaccination, and malaria (an important element to consider in the case of the AIDS epidemic in Africa). Supporting each factor, Johnson provides scientifically valid evidence – published in reputable peer-reviewed journals such as *AIDS, the Proceedings of the National Academy of Sciences of the United States of America, The Lancet, the Canadian Medical Association Journal*, and the *Journal of the American Medical Association (JAMA)* (13).

Celia Farber’s book, Serious Adverse Events: An Uncensored History of AIDS (14) – an exposé of the epidemic’s ethically questionable history – contains an interesting appendix authored by Rodney Richards. Richards – who helped to develop the first ELISA test for HIV – outlines the “evolution” of CDC’s stances regarding the role of antibodies, infection, and HIV tests. First, the CDC aligned itself with the traditional view of antibodies signaling past/prior infection (as evidenced in the quote above, from 1984). In 1986, the CDC moved toward a qualified claim, stating:

… patients with repeatedly reactive screening tests for HTLV-III/LAV antibody … in whom antibody is also identified by the use of supplemental tests (e.g., WB, immunofluorescence assay) should be considered both infected and infective [(15), p. 334].

Finally, in 1987, CDC adopted a non-qualified claim that antibodies signify active infection and/or illness: “The presence of antibody indicates current infection, though many infected persons may have minimal or no clinical evidence of disease for years” [(16, 17), p. 509].

A more specific measure than the ELISA test, the WB detects antibodies by identifying proteins believed to be associated with HIV, and only with HIV. A person undergoes a confirmatory WB after a prior ELISA screening test reacts positively (but it is important to remember: over 60 conditions can yield a false-positive ELISA) (13, 18).

Critics of the orthodox view decry the lack of standardized criteria for a positive result in a WB, across countries, world-wide (19). Bauer (Table 1), in a 2010 article titled “HIV tests are not HIV tests” claims, “no fewer than five different criteria have been used by different groups in the United States” [(18), p.7]. Moreover – adds Bauer – included in the contemporary criteria for a positive WB are p41 and p24, protein–antigens “found in blood platelets of healthy individuals.” This means some of the biological markers being used to “flag” the presence of HIV are not “specific to HIV or AIDS patients [and] p24 and p41 are not even specific to illness.” In other words, healthy persons may test positive on a WB but not carry HIV at all [(18), p. 6].

**Table 1:** **Credentials and professional experience of select critics of the HIV-AIDS hypothesis**.

Name (alphabetical order by last name)	Credentials
Henry Bauer, Ph.D.	Professor Emeritus of Chemistry and Science Studies
	Dean Emeritus of Arts and Sciences
	Virginia Polytechnic Institute and State University (Virginia Tech)
James Chin, MD, MPH^a^	Chief of Infectious Disease Section, California State Department of Health Services, Berkeley, CA, USA (1970s–1987)
	Former Chief of Surveillance, Forecasting and Impact Assessment (SFI), Unit of the Global Program on AIDS (GPA) of the World Health Organization Editor: APHA’s “Control of Communicable Diseases Manual”
Ettiene de Harven, MD	Emeritus Professor of Pathology: University of Toronto, ON, USA
	Specialized in electron microscopy at the “Institute du Cancer” in Paris
	Published first images of budding virus through EM (1960)
	Member: Sloan Kettering Institute, New York, NY, USA in 1968
	Former President: The Electron Microscopy Society of America (in 1976)
	Former President: Rethinking AIDS
Peter Duesberg, Ph.D.	Professor of Molecular and Cell Biology: The University of California, Berkeley, CA, USA
	Isolated the first cancer gene and mapped the genetic structure of retroviruses (1970)
	Member: National Academy of Sciences (since 1986)
	Outstanding Investigator Award – National Institutes of Health 1986
Heinrich Kremer, MD	Founder and Senior Consultant: Cell Symbiosis Therapy Academy^®^ (based on his work on NO and its association with chronic inflammatory and degenerative disease)
	Collaborating Member: Study Group for Nutrition and Immunity (Bern, Germany)
	Extensive clinical work with youth drug addiction
Kary Mullis, Ph.D.	Nobel Laureate – Chemistry – 1993
	Developed: polymerase chain reaction
	Founder and Chief Scientific Advisor: Altermune
David Rasnick, Ph.D.	Biochemist with >25 years of work with proteases and protease inhibitors
	Former President: Rethinking AIDS: the group for the scientific reappraisal of the HIV hypothesis
	Former President: international coalition for medical justice

*^a^ Chin agrees with the mainstream hypothesis that HIV is the cause of AIDS. His critique centers on the collection and interpretation of the epidemiological data for HIV/AIDS, in the US and world-wide*.

An example may clarify: if tested in Africa, a WB showing reactivity to any two of the proteins p160, p120, or p41, would be considered positive for HIV. In Britain, the test would be positive only if it showed reactivity to one of these three proteins, together with reactions to two other proteins, p32 and p24 (see mention of p24, above, as occurring in healthy individuals). Therefore, someone whose test reacts to p160 and p120 would be considered HIV-positive in Africa, but not in Britain. A test reaction to p41, p32, and p24 would be considered positive in Britain, but negative in Africa, leading author Celia Farber to comment: “… a person could revert to being HIV-negative simply by buying a plane ticket from Uganda to Australia [or in our example, from Uganda to London” (14), p. 163].

According to critics, a definitive answer regarding which protein–antigens are specific to HIV and HIV alone can only come from successful virus isolation and purification. Isolating and purifying “would be required to verify that all of these proteins actually originate from HIV particles” [(7), p. 70]. Attempts at purifying have been made (20, 21), but have been criticized for their ambiguous findings (22), or for their use of cultured samples (see discussion below on EM images). To date, the issue of HIV isolation in purified samples has not been addressed to critics’ satisfaction (23).

#### Viral load

The expression “viral load” refers to the quantity of virus found in HIV-infected blood. According to the mainstream perspective, information on viral load helps monitor the infection’s progress, “decide when to start treatment, and determine whether or not … HIV medications are working” (24).

The technique for measuring viral load is known as RNA PCR – ribonucleic acid polymerase chain reaction (25). Mainstream scientists regard this test as the most specific documentation of HIV’s presence in a person’s body. It is often used when the ELISA and WB tests are negative, because PCR can detect the virus’ genetic material (or its RNA/DNA fragments), before the human body has had a chance to recognize the virus, produce antibodies in defense, and react positively in an antibodies-only test (26).

Despite its enhanced specificity, many mainstream scientists and practitioners recommend caution when using PCR for screening or diagnosing infection (27). For instance, authors of a study published in JAMA in 2006, in which PCR was used with a sample of almost 3,000 people, concluded: “The PCR assay is not sufficiently accurate to be used for the diagnosis of HIV infection without confirmation” [(28), p. 803].

PCR technology evolved quickly since it was introduced in 1983 (25). Although being employed, mostly, for assessing viral load (less for screening and diagnosis), it should give us pause to learn, however, that Dr. Kary Mullis – the scientist who won the 1993 Nobel Prize for inventing the PCR test and whose quote introduced this article (Table 1) – has strongly opposed using the technique for determining the amount of virus circulating in plasma. Lauritsen explains:

Kary Mullis … is thoroughly convinced that HIV is not the cause of AIDS. With regard to the viral-load tests, which attempt to use PCR for counting viruses, Mullis has stated: “Quantitative PCR is an oxymoron.” PCR is intended to identify substances qualitatively, but by its very nature is unsuited for estimating numbers. Although there is a common misimpression that the viral-load tests actually count the number of viruses in the blood, these tests cannot detect free, infectious viruses at all; they can only detect proteins that are believed, in some cases wrongly, to be unique to HIV. The tests can detect genetic sequences of viruses, but not viruses themselves [(29), p. 3].

If to this picture we add human endogenous retroviruses (or HERVs) (30) as potential confounders, the genetic sequences detected in a PCR test may not be those from an exogenous virus, at all, and may explain the test’s substantial false-positive rates (18, 27). HERVs consist of retrovirus-like particles produced by host cells that are stressed or dying. In other words, when various infections assail the body, and certain cells experience stress or die in large numbers, they can manufacture by-products similar to retroviruses. These by-products can be reactive when testing for HIV antibodies, protein antigens, and viral loads (31). Culshaw summarizes it well:

A retrovirus is nothing more than RNA with an outer protein shell. The shell enables it to bind to cells of the type it infects, and once it gains entry, the outer coating disappears and the RNA is transcribed to DNA and incorporated as provirus into the host cell’s own genome. It is for this reason that retroviruses are called enveloped viruses, and it is also the reason that it is very difficult to distinguish between exogenous retroviruses (those that originate outside the body from a foreign invader) and endogenous retroviruses (those that are manufactured from our own retroviral-like genetic sequences under conditions of cellular stress, including diseases) … Much of the genetic material attributed to HIV is in fact DNA or RNA from [these] decaying cells (…) Human beings are filled with such endogenous retroviruses [(32), pp. 53, 55–56].

### Transmission electron microscopy images of retroviral particles

Although it seems intuitive that photographing HIV would provide undeniable evidence of its presence in the host’s plasma, the reality is much more complex. Adequately interpreting images obtained through EM is, even for the most skilled scientists, challenging. EM generates highly amplified images of cells and viral particles. An electron-microscope uses “beams of electrons focused by magnetic lenses instead of rays of light” to produce images magnified up to 10,000,000× (a light microscope has difficulty exceeding 2000× magnification) (33).

The first images of what researchers believed to be HIV particles budding out of human cells were published in the journal Science, in 1983, by the French team that co-discovered HIV (headed by Luc A. Montagnier) (34). These images, and the computer graphics based on them, were printed in textbooks and articles discussing AIDS, extensively. Despite their popularity, the images were obtained from a “pre-AIDS” patient (not a patient with AIDS), and the sample furnishing the images had not been purified according to standard procedures (35).

It would be 14 years later, in 1997, when EM images from purified samples were produced (20). Yet another study (22), published simultaneously with these images (in fact, printed as an adjoining article), reported: even purified HIV samples harbor protein particles (called microvesicles), considered to be contaminants. These microvesicles do not disappear during the purifying process. In other words, even when technicians purify HIV samples, certain “cellular proteins bound to non-viral particles (i.e., microvesicles) can copurify with [the] virus,” and appear in the EM images. The question, then, remains: are the EM images seen in these purified samples, pictures of HIV itself, or of other elements/particles? (36).

In 2010, Ettiene de Harven – the scientist who “produced the first electron micrograph of a retrovirus (the Friend leukemia virus)” [(32), p.13] through EM research in 1960 (Table 1) (37) – added to the debate:

All the images of particles supposedly representing HIV and published in scientific as well as in lay publications derive from EM studies of *cell cultures*. They never show HIV particles coming directly from an AIDS patient [(7), p. 70 – emphasis added].

Why is it important to obtain EM images of HIV from AIDS patients, as opposed to images of HIV cultured in a laboratory? According to de Harven, non-viral micoorganisms frequently contaminate cell cultures and show up very easily in EM. It is quite difficult to obtain absolutely pure cell cultures, especially because the culturing process itself – the growth factors added to the culture, such as “T cell lymphocyte growth factor (TCGF), interleukin 2, or corticosteroid hormones” [(23), p. 4] – can introduce potential contaminants. HERVs, for example, are often generated by cells that have been stressed or hyperstimulated to grow in cultures. HIV cultures obtained from patients with AIDS may not require as much stimulation or addition of growth factors, thus resulting in less contaminated, purer cultures.

Montagnier also acknowledges the problems with relying on EM to identify a retrovirus, given the difficulties with purifying viral samples. In an interview given in 1997, he reflects on those first HIV images from cultured samples, produced in his laboratory at the Pasteur Institute:

DT (Djamel Tahi): Why do the EM photographs published by you, come from the culture and not from the purification?

LM (Luc Montagnier): There was so little production of virus it was impossible to see what might be in a concentrate of virus from a gradient. There was not enough virus to do that …

(…)

DT: How is it possible without EM pictures from the purification, to know whether these particles are viral and appertain to a retrovirus, moreover a specific retrovirus?

LM: Well, there were the pictures of the budding. We published images of budding which are characteristic of retroviruses. Having said that, on the morphology alone one could not say it was truly a retrovirus … (38).

It appears, therefore, there is little consensus regarding what the existing EM images reflect: are the visualized particles HIV or something else? According to Papadopulos-Eleopulos and colleagues, “some of the best known retrovirologists including Peter Duesberg, Robert Gallo, and Howard Temin have been telling us that particles may have the morphological characteristics of retroviruses but are not viruses” [(39), p. 2]. It is feasible, therefore, that EM images are, in fact, depictions of (a) microvesicles (or protein particles), not viral or infectious in nature, but not eliminated even when using purified samples (22); or (b) human endogenous retroviruses – defective, non-infectious retroviruses associated with the host’s own genome (see discussion above on HERVS).

### Efficacy of anti-retroviral drugs

From the epidemic’s onset, researchers worked relentlessly to find a vaccine to keep the virus from spreading and to develop drugs for managing the symptoms from opportunistic infections (40). The challenges inherent in developing both vaccine and treatment were daunting: post-infection, HIV appears to mutate and recombine continually, thus making it difficult to design an effective vaccine (41, 42). Furthermore, designing treatments for a retrovirus is a tricky feat, given it shares many of the same characteristics of the host’s immune cells – thus, an attack on the virus can become a simultaneous attack on the healthy host cells (14, 32, 35).

After the public announcement regarding the probable cause of AIDS, various pharmaceutical companies tried to develop drugs to thwart the action of the virus’ reverse transcriptase enzyme (an enzyme essential for the replication of retroviruses). AZT became the first medication of this kind, approved specifically for treating AIDS patients in 1987 (43). Azidothymidine (AZT) – also known as Retrovir, a drug originally designed, but proven unsuccessful, for treating leukemia – made history not only because it was the first available treatment specifically for AIDS, but also due to how quickly it was approved: AZT received “investigational new drug (IND) status (initial approval for testing) within 5 days of application” [(44), p. 134]. Given the desperate need for specific treatment, the drug’s placebo-controlled trials also moved fast, lasting “only 6 months before approval was given for general sale” [(44), p. 134]. Phase II trials were interrupted, mid-way, due to findings that fewer patients taking AZT were dying of AIDS when compared to the control group not taking the drug (44, 45).

Approving AZT, however, did not prevent scientists from trying to develop other drugs, during the following decade; but most attempts would make little headway into the treatment of AIDS. Adding to these difficulties, AZT was proving to be extremely toxic and not as effective as initially anticipated. Researchers did learn, meanwhile, that prescribing AZT in lower dosages and in combination with other, well-known drugs such as heparin, acyclovir, and bactrim, was beginning to curb mortality rates (44).

Thus, in the mid-90s “combination therapy” became available. Also referred to as the “drug cocktail,” combination therapy comprised a joint attack on HIV using three main classes of drugs, simultaneously: (a) those inhibiting reverse transcriptase’s ability to duplicate the virus’ genetic material using host DNA sub-divided into two classes – nucleoside and non-nucleoside inhibitors; (b) protease inhibitors (designed to limit certain proteins needed for HIV assembly); and (c) myristoylation or entry/fusion inhibitors (blocking the virus from entering the host cells). These three classes of drugs – known collectively as HAART (highly active ARV therapy) or antiretrovirals (ARVs) – have been praised for their ability to restore the health of patients with AIDS who become extremely ill [(24, 44, 46), p. 240].

Antiretrovirals also are praised for their ability to reduce patients’ viral loads and, therefore, their level of infection and ability to transmit the virus (or infectivity). This reduction in viral load has been deemed so significant that, in 2012, the FDA approved using one of the combination drugs (Truvada) for pre-exposure prophylaxis or PrEP (47).

PrEP or “HIV treatment-as-prevention” (48) involves administering to non-infected persons one pill of the antiretroviral, daily, to stave off infection: an initiative crowned *Breakthrough of the Year* by the journal Science, in 2011 (47). Trials conducted world-wide have consistently demonstrated low rates of HIV infection among people taking PrEP (41, 48). The 2011 breakthrough, therefore, was the conclusion: “The early initiation of ARV therapy reduced rates of sexual transmission of HIV-1 and clinical events, indicating both personal and public health benefits from such therapy” [(41), p. 493].

Yet, as with most treatment drugs, ARVs also produce important side-effects. Even mainstream scientists who praise the drugs by saying, “Combination theory [*sic*] was a miracle, comparable with antibiotics, anesthesia, and the polio vaccine in the annals of the history of medicine … a ‘quantum leap”’ – candidly admit: “The miracle was not without complications.” [(44), pp. 246, 247]. Because these drugs also attack non-infected cells, they can destroy the immune systems’ healthy T-cells, and even cause a collapse identical to AIDS. Authors of a study reporting on the first decade of ARV use concluded,

The results of this collaborative study, which involved 12 prospective cohorts and over 20,000 patients with HIV-1 from Europe and North America, show that the virological response after starting HAART has improved steadily since 1996. However, there was no corresponding decrease in the rates of AIDS, or death, up to 1 year of follow-up. Conversely, there was some evidence for an *increase in the rate of AIDS* in the most recent period [2002–2003] [(49), p. 454 – emphasis mine].

Critics’ concerns center on the potential association between use of HAART and a depressed immune system. This association carries significant implications for the prophylactic use of ARVs. For instance, studies have documented patients’ compromised immune systems as *preceding* their seroconversion (50, 51). Therefore, having non-infected persons take HAART as prophylaxis may, over time, impact their immune systems negatively, and predispose them to becoming infected with various agents, including HIV itself. Moreover, there is evidence that ARVs can accelerate aging of cells in ways that promote progressive multi-organ disease (52). Critics also point to data on patients taking ARVs who develop *Pneumocystis Carinii*, and *Candida albicans* (opportunistic infections typical of patients with AIDS) while on the drugs, despite the fact the protease inhibitors have “marked anticandidal and antipneumocystis effects” [(7), p. 71]. Equally vexing, are the deaths among ARV-treated patients, resulting from acute liver failure. These deaths point to the ARVs’ detrimental effects, given that HIV, itself, does not cause liver toxicity (7, 53, 54).

Critics also highlight studies documenting the reduction of plasma HIV RNA among patients treated with ARVs, but the non-reduction in HIV DNA, suggesting there is “continued expression of viral agents” even after 1 year of treatment [(55), p. 320]. Compounding these difficulties are the often debilitating side effects (45), the drugs’ extremely high costs (AZT alone cost around $6,000 a year and the cocktails can easily tally $12,000 – 13,000 a year per patient) [(44), pp. 245–246] and the oftentimes daunting regimen some prescriptions require, leading to patients’ less-than-optimal compliance during treatment.

Despite this host of problems, orthodox scientists and practitioners still claim HAART has changed the face of the AIDS epidemic: once considered a lethal syndrome, testing positive for HIV does not equate to a death sentence any longer; merely to a lifetime of managing a chronic infection (56, 57). Critics, on the other hand, assert: because the drugs are anti-viral and anti-bacterial in nature, they give a false impression of being effective for treating HIV infection. What appears a miraculous recovery in many patients is, in fact, the drugs’ effects upon the opportunistic infectious agents the person may harbor at the time, other than HIV. Contrary to the reigning enthusiasm for ARVs’ effectiveness for prevention and treatment, critics will argue the risks associated with ARVs appear to outweigh the benefits, especially if these drugs are consumed over long periods of time. In short, unorthodox scholars believe the appearance of effectiveness of ARVs does not represent strong evidence for the role of HIV in AIDS and, in a paradoxical manner; ARVs may actually be the cause of AIDS-defining illnesses and non-AIDS-defining ones.

### Epidemiological data

It is easy to obtain current statistics describing the HIV-AIDS distribution, world-wide. One has only to access the website of the Joint United Nations Program on HIV to learn: “In 2012, there were 35.3 million [32.2–38.8 million] people living with HIV” and that, in the same year, “1.6 million [1.4–1.9 million] people died from AIDS-related causes worldwide compared to 2.3 million [2.1–2.6 million] in 2005” (58).

Scholars on both sides of the debate agree: “epidemiologic studies and data can show only that a risk factor is statistically associated (correlated) with a higher disease incidence in the population exposed to that risk factor” [(59), p. 42]. Epidemiological data do not provide evidence for causation. All the data can do is reveal risk factors and illness co-occurring in a given group. Despite this well-known caveat, mainstream scientists argue that because HIV has spread among high-risk groups as expected, the AIDS epidemic has, indeed, a viral, infectious agent: its “epidemic curves resemble … such infectious agents as hepatitis B and genital herpes viruses” [(59), p. 53]. These scientists also will explain the differences observed in the frequency of certain illness in specific geographic regions (e.g., higher numbers of HIV-related Tuberculosis in sub-Saharan Africa) as caused by the “background flora of infectious disease agents” present in these regions [(59), p. 54].

Curiously, however, even among mainstream scholars who believe epidemiological data constitute valuable evidence of a viral cause for AIDS, there are those who have turned a critical eye toward the data the US and the WHO have compiled. James Chin – one such critic (Table 1) writes in his book, *The AIDS Pandemic: The Collision of Epidemiology with Political Correctness*:

Estimation and projection of HIV infections and AIDS cases and deaths (HIV/AIDS) can be considered more of an art than a science because of the marked limitations of both available data and methods for estimation and projection. These limitations make it possible for UNAIDS and other AIDS program advocates and activists to issue misleading and inflated estimates and projections [(59), p. 137].

The questions regarding the validity and reliability of epidemiological data emerging from within the mainstream/orthodox views have been echoed and amplified by unorthodox scholars. Both camps’ concerns center on four problems plaguing the estimates of incidence (new cases), prevalence (remaining cases), and projection (future cases) of HIV infections, AIDS diagnoses, and AIDS-related deaths: (a) the varying clinical definitions of AIDS (the official definition has changed four times since 1982) (60); (b) variability in the criteria for seropositivity in HIV tests; (c) the absence of testing in many regions of the world (many developing countries do not have the laboratories needed to test every single AIDS case); and (d) the mistakes in estimation, data management and reporting (e.g., the revision of projections for year 2006 by UNAIDS) (59–62).

This article’s space limitations do not allow an expanded treatment of each problem-area, but readers can find further details within the works cited. For instance, in Rebecca Culshaw’s book – *Science Sold Out: Does HIV Really Cause AIDS* (32) – readers will find 13 “failed predictions” regarding the spread of HIV and AIDS, including the prediction that HIV infection would spread randomly among populations (i.e., outside specific risk groups). Culshaw also tells her personal story of having written a master’s thesis, received a Ph.D. based on her work with “mathematical models of the immunological aspects of HIV infection,” and eventually concluding “there is good evidence that the entire basis for this theory is wrong” [(32), p.7].

## Unorthodox Theories: If not HIV, Then What?

If the criticisms outlined above pinpoint significant problems with each type of data used to support the HIV-AIDS hypothesis, they only contribute to deconstructing the hypothesis, not to providing explanations for what might cause AIDS if not a retrovirus. However, alternative hypotheses abound. Anchoring themselves in well-established causes of immune system malfunction, these hypotheses point to pharmacological (drug) factors, immune dis-balance factors, latent infection overload, and malnutrition as culprits.

Although several scientists investigated the role drugs might play in causing immune suppression *before* HIV was identified [see a list of these studies in Duesberg et al. (46)], the main proponent of the drug-AIDS hypothesis in the epidemic’s early years was Peter Duesberg, a professor of Molecular and Cell Biology at UC Berkeley. According to Seth Kalichman, who wrote *Denying AIDS* (a harsh critique of unorthodox views and of Duesberg in particular), “In every respect, HIV/AIDS denialism starts and ends with Peter Duesberg” [(63), p. 175]. Duesberg’s arguments gained notoriety among unorthodox theories not only due to his expertise and prominence (see Table 1), but also to his challenge of the medical and scientific establishments early in the history of the epidemic, employing clear empirical logic.

Duesberg began challenging the viral hypothesis for AIDS soon after the publication (in 1984) of the four seminal articles pointing to HIV as the “probable” cause (64–67). In two key publications in 1987 and 1989 – in *Cancer Research* and in the *Proceedings of the National Academy of Sciences* (68, 69) – Duesberg cogently argued: retroviruses are not known for killing cells. In other words, retroviruses are not “cytocidal.” If anything, retroviruses were once thought to be associated with cancer because they cause precisely the opposite of cell death; they contribute to cells’ growth or proliferation. In Duesberg’s words, “… retroviruses are … considered to be plausible natural carcinogens because they are not cytocidal and hence compatible with neoplastic growth and other slow diseases.” [(68), p. 1200]. In his view, HIV’s inability to kill cells could not explain the suppression of the T-cells in the immune system, as proposed by the teams who discovered HIV^3^. According to Farber,

In other fields, such as gene therapy, it is axiomatic that retroviruses are the ideal carriers for genetic materials, because they ‘don’t kill cells’. Incredibly, this is where the so-called HIV debate first forked in 1987, and where the camps remain bitterly divided to this day [(14), p. 50].

For Duesberg and scientists agreeing with him, then, other agents would have to be responsible for the disastrous immune function collapse seen in AIDS patients. These scientists saw as prominent among such causes, the use of drugs, both recreational and routinely prescribed ones. As author Gary Null points out, even before AIDS, researchers were documenting the immune-suppressing effects of amyl nitrites or “poppers” (the form of amyl nitrites popular among gay men in the early and mid-80s) and determining both their toxicity and carcinogenic properties in humans and animals (45). However, two studies CDC published in 1983, one in which they were unable to detect any toxicity from amyl nitrites, the other, unable to document a significant association between inhaled nitrates and Kaposi’s sarcoma or *Pneumocystis carinii* pneumonia, led the search to a halt (70, 71). Investigators later tried to determine if certain *batches* might have been contaminated with toxic agents but, when they found no contamination, the focus on poppers/amyl nitrites themselves ceased (1). Nonetheless, in 1998 Duesberg and Rasnick (Table 1) (72) reviewed evidence published since 1909, “which prove[s] that regular consumption of illicit recreational drugs causes all AIDS-defining and additional drug-specific diseases at time and dose-dependent rates” [(46), p. 393].

Other drugs such as those given to transplant patients to prevent organ rejection, as well as routinely prescribed antibiotics, also have been implicated as potential causes of immune dysfunction. Studies have shown that transplant patients who develop Kaposi’s sarcoma will go into remission, once taken off the drugs required to avoid organ rejection. Immune-suppressing drugs (as well as amyl nitrites) have, for instance, been directly correlated with Kaposi’s sarcoma, the rare skin cancer found frequently among AIDS patients during the epidemics’ early days [see reviews by Null (45) and Kremer (35)].

Anti-retroviral drugs used to treat HIV infection/disease, also, are indicted by Duesberg and those who agree with him as potentially causing AIDS (43, 62). Because the drug cocktails include “DNA chain-terminators and protease inhibitors” that affect healthy cells as well as the virus, and because “many studies find that people receiving ARV medications experience AIDS-defining diseases to a greater extent than controls not receiving those medications” [(73), p. 122], antiretrovirals are viewed as potential immune suppressors.

In a review of the chemical bases for AIDS, published in 2003, Duesberg and his colleagues (46) outlined the epidemiological and bio-chemical evidence supporting different causes for the AIDS epidemics in the US/Europe and in Africa, none of which are viral or contagious. The authors concluded:

The chemical-AIDS hypothesis proposes that the AIDS epidemics of the US and Europe are caused by recreational drugs, alias lifestyle, and anti-HIV drugs … and by other non-contagious risk factors such as immunosuppressive proteins associated with transfusions of blood clotting factors … pediatric AIDS is due to prenatal consumption of recreational and anti-HIV drugs by unborn babies together with their pregnant mothers … The chemical basis of African AIDS is proposed to be malnutrition and lack of drinkable water … exactly as proposed originally by the now leading HIV-AIDS researchers Fauci and Seligman: “The commonest cause of T-cell immunodeficiency worldwide is protein-calorie malnutrition” … and others … [(46), p. 392].

Alongside a drug hypothesis, another proposed cause for AIDS is the iNOS hypothesis, or immune dis-balance hypothesis. In his book, *The Silent Revolution in Cancer and AIDS Medicine*, Kremer (35) (Table 1) explains that much of what scientists now know about the immune system and its functions was not well understood at the time they identified HIV. In particular, the research on NO, or nitric oxide, was still in its infancy: NO is “an important intracellular and intercellular signaling molecule” acting as “…an important host defense effector in the immune system” [(74), p. 639]. Even though NO (and its derivative iNOs) is “involved in the regulation of diverse physiological and pathophysiological mechanisms in cardiovascular, nervous, and immunological systems,” researchers have shown it can also become a harmful, “cytotoxic agent in pathological processes, particularly in inflammatory disorders” [(74), pp. 639–640]. Put simply, at adequate levels NO helps regulate blood pressure as well as “wound repair and host defense [*sic*] mechanisms” [(75), p. 277]. Excessive amounts, however, lead to T-cell depletion, “inflammation, infection, neoplastic diseases [cancer] liver cirrhosis, [and diabetes” [(75), p. 277]. This change from adequate-to-excessive amounts of NO in the human body results from multiple factors, including “nitrite inhalation [e.g., using ‘poppers’], microbial antigen, and toxin stimulation [e.g., suffering repeated infections with different viruses/bacteria], immunotoxic medications [e.g., taking ARVs and antibiotics], [and] many other stress factors” [(35), p. 49].

A closely related perspective, placing the blame for AIDS on bio-chemical processes gone awry within human cells is the oxidative stress (or redox) hypothesis. Oxidative stress is a cellular-level electro-chemical phenomenon that diminishes a cell’s ability to absorb oxygen. This diminished capacity to process oxygen at optimal levels leads to the cell’s disruption and death. Scientists have either hypothesized or empirically connected oxidative stress to many diseases, including type 2 diabetes and cancer (35, 45, 76). According to this hypothesis’ main proponents,

At first sight it appears that there is no common factor, apart from HIV infection, linking the various AIDS risk groups. However, homosexuals are exposed to relatively high levels of nitrites and anally deposited sperm, drug abusers to opiates and nitrites, hemophiliacs to factor VIII. All these are known potent *oxidizing agents* … [(77), p. 147 – emphasis mine].

For these proponents of the redox hypothesis even Luc Montagnier (the head of the French team that discovered HIV) agrees “that anti-oxidants should be used for treatment of HIV/AIDS patients” [(78, 79), p. 6].

Viewing a person’s immune system as a complex dynamic balancing act among various elements, which sometimes behave as defenders, other times, as offenders, is also consistent with the “latent infection overload hypothesis” proposed by Kary Mullis (Table 1). According to Mullis, as people become infected with multiple viruses and experience many latent infections, the immune system embarks on a chain-reaction-response to each virus. Latent infections are those without visible symptoms, and according to Mullis, “at a given time most viral infections in an individual are latent” [(80), p. 196]. Eventually, the system overloads itself and becomes dysfunctional. AIDS, he says, “may be the result of such a chain reaction.” This hypothesis assumes:

… there is not a single organism that is the cause of AIDS, and there should exist AIDS patients who do not test positive for HIV^4^ . It is an overwhelming number of distinct organisms, which causes the immune dysfunction. These may individually be harmless [(80), p. 197].

Perhaps the most intriguing alternative hypothesis, however – if not from its bio-chemical perspective, at least from the perspective of who supports it – is the one proposing HIV may not be the primary villain, but merely an accomplice in causing AIDS (83). Joseph Sonnabend – a prominent physician/researcher responsible for encouraging his gay patients to lead a healthy lifestyle to avoid developing AIDS, and one who “did not accept HIV = ADS theory for many years” – recently changed his views and “has come to think that HIV, together with other factors, may play a subsidiary causative role” [(73, 84), p. 120]. Even Montagnier and Gallo (leaders of the French and American teams, respectively, that discovered HIV), at various times since the epidemic began, have suggested HIV might be a co-factor in AIDS, not its exclusive causative agent (85).

Other hypotheses have been proposed over the years, but none have garnered as much attention as those outlined above. Some of these other hypotheses claim AIDS is caused by (a) multiple factors; some factors explaining some cases, other factors accounting for other cases; (b) undiagnosed or untreated syphilis infection; (c) autoimmunity; (d) selenium deficiency, and (e) psychological factors, including stress and trauma [see Bauer (73), pp. 124, 136–139 for details on these hypotheses].

The positive or reassuring aspect of these alternative hypotheses is the tangible hope for prevention, treatment, and cure they embody. Nevertheless, it is difficult not to agree with Bauer when he concludes, “…it is hardly reassuring that this array of suggestions has been in circulation for something like (three) decades without having been adequately explored” [(73), p. 139].

## Discussion

At this point, readers might be wondering: given the problems with the mainstream hypothesis, how did we get here? How did we come so far, tethered to such a problematic perspective? The complexity of the answers to these questions aside, it may help to bear in mind the notion that HIV-causes-AIDS emerged and developed within a very specific scientific-cultural-historic context. Although the scope of this article precludes dealing with this complex context, for our purposes it is important to recall at least one element: Funding for President Nixon’s War on Cancer campaign ended in 1981 with very little achieved in the quest for an infectious cancer agent (15, 85–87). The only exception was the discovery connecting select retroviruses to a few, rare cancers. Other than this, scientists had a handful of “orphaned” viruses which, they suspected, might play a role in causing illnesses, but no known diseases to which these viruses could be connected. Proposing a connection between an emerging syndrome and one of these viruses (even if only a circumstantial connection) proved enticing enough to pursue. And pursue they did, as soon as AIDS began to appear in larger-than-expected numbers among otherwise healthy adults.

If viewed from this perspective, then, why scientists so quickly and assuredly “jumped on the HIV bandwagon” may not be very difficult to understand. That the scientific establishment world-wide insistently refuses to re-examine the HIV-AIDS hypothesis, however, is more difficult to accept, especially when one examines the credentials of those proposing such a revision. Their expertise carries as much weight as the teams who defend the orthodox hypothesis (Table 1). Seth Kalichman, a critic of AIDS “denialists,” recommends adamantly: anyone who entertains alternative views should “consider the source: credibility of where the article is reported as well as the researchers themselves must be weighed” [(63), p. 159]. I could not agree more: taking into account the credibility of the scholars who question the HIV-AIDS hypothesis is, perhaps, the strongest argument *in favor* of seriously considering their critiques, not against it.

Furthermore, credibility as an argument works both ways: if to question the trustworthiness of unorthodox scholars is vital, it is equally crucial to question the reliability of those supporting the HIV-AIDS hypothesis. Readers who care to learn about HIV-AIDS’ history will encounter ethically questionable actions carried out by some of the most notable orthodox researchers, as well as ethical misconduct charges made against them [for an extensive treatment of these ethical and legal issues, backed by extensive official documentation, see Crewdson (88)].

If it is difficult to dismiss the unorthodox views due to the credibility of their sources, then, why are not orthodox scientists and practitioners more willing to rethink the hypothesis or, at the very least, test the unorthodox arguments in a scientific, open debate? Although there have been, in fact, several attempts to engage the orthodox community in dialog, nearly all have been unsuccessful [for examples, see Ref. (14, 85, 88)]. Most likely, reasons for denying the calls to re-examine the orthodox stance lie in the complex, synergistic dynamics within the scientific, medical, economic, and political systems or ideologies worldwide. Even brief speculation about these reasons would exceed the scope of this article, therefore I refer the reader, once again, to the sources referenced [in particular, see Epstein (89) and Bauer (73)].

Here I would argue, nonetheless, that the debate between orthodox and unorthodox scientists comprises much more than an intellectual pursuit or a scientific skirmish: it is a matter of life-and-death. It is a matter of justice. Millions of lives, worldwide, have been and will be significantly affected by an HIV or AIDS diagnosis. If we – the public health workforce – lose sight of the social justice implications and the magnitude of the effect, we lose “the very purpose of our mission” [(3, 90), p. 690].

In particular, a pressing concern for public health is the move or push toward (a) HIV screening for “patients in all health-care settings” (with opt-out screening) (91) and (b) placing persons-at-risk (even if not yet infected with HIV), on retroviral medication as a form of prophylaxis (see discussion about PrEP, above) (92). If in 1986 the CDC recommended voluntary testing for people in high-risk groups, in 2013 the U.S. Preventive Services Task Force “gave routine HIV screening of all adolescents and adults, ages 15–65, an ‘A’ rating” [(93), p. 1]. The recently approved Affordable Care ACT “requires or incentivizes new private health plans, Medicare, and Medicaid to provide preventive services rated ‘A’ or ‘B’ at no cost to patients” [(93), p. 1]. Thus, routine screening of every adolescent and adult in all populations is, now, the goal (91, 94).

If, to this goal we juxtapose the problems with the HIV tests, with the definition(s) of AIDS, and with the toxicity of the ARVs currently prescribed, we begin to understand the potential for harm inherent in them. Put blatantly: these recommendations can be harmful or iatrogenic (95).

### Public health workforce: Our role

What can the public health workforce do, given such potential for harm? As stated in the introduction, this paper represents a call to reflect upon our public health practice vis-à-vis HIV-AIDS. Reflecting upon and questioning the *status quo* constitute important dimensions of public health professionals’ competencies and practice. If the only hope the HIV-AIDS hypothesis can offer, 30 years later, is to provide highly toxic drugs to treat HIV infection and to prevent high-risk but healthy persons from becoming infected, health promoters have a professional duty to reflect on the available data and question the usefulness of the hypothesis. Only in doing so can public health professionals maintain their professional integrity, tend to public health’s roots in social justice, and contribute to developing knowledge using ethical methods.

James Jones, in his book *Bad Blood: The Tuskegee Syphilis Experiment* (96), reminds us poignantly that not asking whether health professionals “should be doing” something, but continuing to do it uncritically, because “it can be done” was, ultimately, the mind-set sustaining the Tuskegee syphilis study for 40 years – unquestionably one of the worst cases of scientific misconduct in American history. The AIDS epidemic – if managed without questioning or without the dialogical process of action-reflection – may, with time, overshadow Tuskegee in the magnitude of its negative impact.

Specifically, I propose the public health workforce can undertake such an action-reflection process by engaging in the following tasks:

(1) Learning about the history of the HIV/AIDS epidemic, of the problems surrounding the discovery of HIV, and about the development of drug therapies and PrEP. Publications recording this history abound in the professional and trade literatures, representing both mainstream and unorthodox view-points. To understand the forces shaping the HIV/AIDS epidemic, we currently experience represents a crucial responsibility of a competent and ethics-driven workforce.
(2) Conducting its own research to test alternative theories for the cause(s) of AIDS and/or to portray the inconsistencies and contradictions in the orthodox hypothesis. Qualitative inquiry, for instance, exploring unorthodox views and the practices of providers, patients, and scientists, might be a fruitful option for challenging prevailing assumptions.
(3) Fostering and mediating a debate among HIV-infected persons, scientists, and health-care providers, to critically assess current beliefs and practices. Public health professionals – who are well-informed about the orthodox and unorthodox perspectives’ strengths and weaknesses – could play an important role as facilitators in this much-needed dialog.

Although carrying out the tasks outlined above may represent a novelty for many public health professionals, for the scientists, practitioners, and investigators who believe a viral hypothesis for AIDS is unproductive, none of this is new. They have combed historical documents (or played a role in the history, themselves); they have amassed substantial amounts of data, and they have made numerous calls for debate. They have held to their beliefs, steadfastly, for the past 30 years. Twenty four years after the first article challenging HIV, Duesberg and colleagues, for instance, still claimed HIV is only a “passenger virus” (one “not sufficient and not necessary to cause a disease”) [(62), p. 81]. While not all unorthodox scholars agree with Duesberg, most still actively defend their critiques of the HIV-AIDS hypothesis and persist in their questioning. As we face the next decade with AIDS still rampant, then, it becomes vital that public health professionals attend to the debate and embark in a questioning of their own.

## Conflict of Interest Statement

The author declares that the research was conducted in the absence of any commercial or financial relationships that could be construed as a potential conflict of interest.

## Footnotes

^1^In this article, I will use the terms unorthodox, non-orthodox, non-mainstream, and alternative, to refer collectively to those who disagree with the prevalent view, and to their propositions (despite their variability). I will favor the term “unorthodox” for it carries the notion of intention or willful deviation from the norm and connotes a power differential in which one set of theories (the orthodox or mainstream) dominates another – what Delborne calls “the epistemological tyranny of the intellectual majority” [(2), p. 510].

^2^I am indebted to E. de Harven (7) for suggesting these categories.

^3^In fact, evidence supporting the notion “HIV kills T-cells” has been so conspicuously absent that, currently, scientists don’t believe HIV “kills T-cells in any way. Rather, they believe HIV primes T-cells to commit suicide at some later time” [(32), p. 73]

^4^Some would argue this is the strongest evidence against the HIV-AIDS hypothesis: cases of AIDS with no documentable presence of HIV. However, say the critics, the difficulty with this argument lies in the definition of AIDS: because AIDS is defined as “the final stage of HIV infection” (81), AIDS presupposes infection with HIV, making the definition a circular one (i.e., AIDS = final stage of HIV infection = opportunistic infections + high viral load + low CD_4_ counts). Due to the circularity in the logic, if there is no HIV, there can be no AIDS. Nonetheless, cases of patients with AIDS-defining opportunistic infections and low CD_4_ counts without HIV do exist (see, for example, the review by Green and colleagues (82).
